This article has been retracted.

# Intervention Value of Path-Type Health Education on Cognition and Renal Function of Patients with Diabetic Nephropathy

**DOI:** 10.1155/2021/3665460

**Published:** 2021-12-22

**Authors:** Lianfang Bao

**Affiliations:** Department of Outpatient, The First People's Hospital of Fuyang Hangzhou, Hangzhou, 311400 Zhejiang, China

## Abstract

**Objective:**

Analyze and examine the effectiveness of path-based health education for patients with diabetic nephropathy and renal function.

**Methods:**

The 162 diabetic nephropathy patients admitted to our hospital from January 2018 to January 2021 were selected, and participants were randomly assigned to groups: study group (*n* = 79) and control group (*n* = 83). The control group received routine nursing care, whereas the study group received path-type health education. GQOLI-74, MUIS-A scores, biochemical indicators, dietary indicators, cognition, blood glucose levels, and renal function were compared between the two groups.

**Results:**

The GQOLI-74 score of the two groups was substantially higher, while the MUIS-A score was significantly lower, although the study group changed more significantly (*P* < 0.05) than the control group. The biochemical markers in both groups decreased significantly, but the study group changed more dramatically (*P*0.05) than the control group; the nutritional index values of both groups increased significantly, but the study group's nutritional index values increased significantly (*P*0.05) when compared to those of the control group; the control group's awareness of drug treatment, basic knowledge, exercise, and diet was 79.4 percent, 78.9 percent, 73.4 percent, and 91.0 percent, respectively, and the study group's awareness of drug treatment, basic knowledge, exercise, and diet was 90.3%, 96.4%, 92.8%, and 94.0%. The study group exhibited greater awareness (*P*0.05) than the control group. The blood glucose indices of both groups were dramatically lowered; however, the study group's blood glucose level declined more significantly (*P*0.05) than the control group. The renal function indices of both groups were considerably lower, but the study group's renal function indexes were significantly lower (*P*0.05) than those of the control group.

**Conclusion:**

Pathway health education is a new nursing method that can adjust nutritional indicators, improve blood sugar and kidney function, and significantly increase patients' awareness of the disease, which can further improve patient compliance with treatment. This nursing method has high application feasibility and high clinical value.

## 1. Introduction

Diabetic nephropathy is a prevalent condition that severely limits patients' capacity to work and live normally. Active clinical treatment and partnership with intervention should be adopted to reduce the occurrence of end-stage renal disease [1]. Patients with diabetes are more likely to develop nephropathy, which activates the mesangial cells of glomerular cells, causing significant alterations in biochemical indicators such as albumin and proteinuria, which are not conducive to better liver and kidney function [2]. In clinical practice, hypoglycemic medications are often utilized. Some scholars have pointed out that combining nursing intervention based on treatment has more significant effects.

The study selected 162 diabetic nephropathy patients admitted to our hospital from January 2018 to January 2021and carried out routine care and path-based health education to the patients, respectively, and the value of path-based health education around the awareness of diabetic nephropathy patients and renal function intervention. The analysis hopes to improve the various biochemical indicators and speed up the recovery of the disease. The relevant content is now reported as follows.

## 2. Materials and Methods

### 2.1. Data

Between January 2018 and January 2021, 162 diabetic nephropathy patients were hospitalised to our hospital and randomly assigned to one of two groups: the study group or the control group. The study group (*n* = 79), 42 males and 37 females, had a disease duration of 1-13 years, an average of 6.72.2 years, an age range of 30-85 years, and an average age of 65.43.5 years; the control group (*n* = 83), 42 males and 41 females, had a disease duration of 1-13 years, an average of 6.82.4 years, an age range of 30-85 years, and an average age of 65.53.6 years. The findings are similar (*P* > 0.05), the patient is informed of the research, and the hospital's ethical committee has authorised the study.

Criteria for inclusion are as follows [3]: (1) those who satisfy the diagnostic criteria for diabetic nephropathy; (2) those with full clinical data, normal cognitive function, and written informed consent; (3) those who are eligible for prognosis follow-up; and (4) those with stable vital signs. (1) Patients with different kidney problems, such as glomerulonephritis and urinary tract infection; (2) patients who used medications that impair cardiac function throughout the trial time; (3) patients with mental illness; and (4) patients with diabetic ketoacidosis were excluded from the study.

### 2.2. Methods

Routine nursing: preach and educate about diabetes-related knowledge and issues, as well as reply to patient questions. The educational content, methods, and goals are not all the same. Routine interventions, such as medication counseling, life support, and the distribution of health manuals, are also carried out. Path-type health education: (1) establish a nursing team, refer to relevant materials and literature, and combine with the actual situation of the hospital to make a health education path table, including disease prevention, etiology, lifestyle, and other related content. Complete relevant content such as discharge guidance, admission assessment, blood glucose monitoring, rehabilitation guidance, diet and exercise guidance; implement and set intervention measures according to the path table; and intervene through model preaching, concentrated lectures, health manuals, one-to-one explanations, etc. Actively evaluate the effect of the intervention and analyze the patient's knowledge mastery. (2) Diet intervention: evaluate energy according to the patient's body mass; classify food sodium content, calories, and protein. Do not eat high-salt, high-protein, and high-sugar foods. Consume more fatty acid-rich, high-quality, low-protein, and low-cholesterol meals, and treat trace elements and vitamins on a regular basis. To guarantee that the patient's diet is suitable, supplement and match meals according to one's nutritional level. (3) Psychological intervention: fully comprehend personal traits, information, social background, and family; provide adequate care to patients; develop a positive nurse-patient connection; and build trust. Understanding the patient's mental state, actively appraising, improving communication, thinking about difficulties from a new viewpoint, and comprehending the patient's inner sentiments will all aid in the release of negative emotions. (4) Perform relaxation training, such as muscle training and breathing coaching, according to the patient's tolerance and recovery state to manage negative emotions and calm the body and mind.

### 2.3. Outcome Measurement

#### 2.3.1. GQOLI-74 and MUIS-A Score [4]

The comprehensive quality of life assessment questionnaire (GQOLI-74) was used to evaluate the quality of life of patients. There were 74 items, 20 factors, and 4 dimensions in total. The psychological, social, physical, and life functions were evaluated separately. The lower the score, the lower the quality of life and the more serious the impact. The MUIS-A scale is used to evaluate the uncertainty of the disease. It contains 32 items such as ambiguity, complexity, inconsistency, and unpredictability. The Likert 5-level scoring method is used for evaluation. A score of 5-1 indicates complete agreement to complete disagreement. There are 32 items in total. The lower the score, the less the uncertainty about the disease.

#### 2.3.2. Biochemical Indicators [5]

Take 3 ml of fasting venous blood, centrifuge it at a speed of 3500 rpm for a total of 10 minutes, and store it at -80°C. The enzyme-linked immunosorbent test was used to detect changes in total cholesterol, triglycerides, and urea nitrogen levels, and the procedures were followed to the letter.

Transferrin (TRF), serum albumin (PA), albumin (ALB), and other markers are included in the nutrition index.

Medication, fundamental knowledge, exercise, food, and other components of cognition are all included in this perspective. Blood sugar level [6]: the blood glucose analyzer was used to detect the blood glucose (2hPG) and fasting blood glucose (FPG) levels of 2 h after a meal.

Kidney function: urea nitrogen (BUN) and serum creatinine (Scr) are two indicators; the more the value tends to the normal value, the better the intervention effect.

#### 2.3.3. Statistical Techniques

The statistical data was evaluated using the SPSS 19.0 statistical program, and the statistical data was checked using a two-sided test. *P* < 0.05 indicates that the difference is statistically significant; quantitative data is represented by (*xs*), data is compared using the *t*-test, analysis of variance is used to compare three groups of samples, the results are compared using LSD pairwise, qualitative data is compared using the *χ*^2^ test, and the graph is created using GraphPad Prism 8, and the difference is obvious when *P*0.05 is used.

## 3. Results

### 3.1. Comparison of GQOLI-74 and MUIS-A Scores between the Two Groups before and after Nursing

Before nursing, there was no significant difference in GQOLI-74 and MUIS-A scores between the two groups (*P* > 0.05). After nursing, the GQOLI-74 of the two groups was significantly increased, and the MUIS-A score was significantly reduced. But compared with the control group, the study group has more obvious changes, and the difference is statistically significant (*P* < 0.05), as shown in Table 1.

### 3.2. Changes of Biochemical Indicators before and after Nursing in the Two Groups

There was no significant difference in indicators such as total cholesterol, triglycerides, and urea nitrogen between the two groups (*P* > 0.05). After nursing, the biochemical indicators of the two groups decreased significantly, but compared with the control group and the study group, the changes were more obvious, and the difference was statistically significant (*P* < 0.05), as shown in Table 2.

### 3.3. Comparison of Nutritional Indicators between the Two Groups before Nursing

There was no significant difference in ALB, PA, TRF, DPI, mPCR, and other nutritional indicators between the two groups (*P* > 0.05). After nursing, the nutritional index values of the two groups increased significantly. However, compared with the control group, the nutritional index values of the study group increased more significantly, and the difference was statistically significant (*P* < 0.05), as shown in Figure 1.

### 3.4. Comparison of Cognition between the Two Groups before and after Nursing

The control group's awareness of drug treatment, basic knowledge, exercise, and diet was 79.4%, 78.9%, 73.4%, and 91.0%, respectively, and that of the study group was 90.3%, 96.4%, 92.8%, and 94.0%. Compared with the control group, the study group had higher awareness (*P* < 0.05), as shown in Figure 2.

### 3.5. Changes of Blood Glucose Levels in the Two Groups before and after Nursing

Before nursing, there was no significant difference in blood glucose indexes of FPG and 2hPG between the two groups (*P* > 0.05). After nursing, the blood glucose indexes of the two groups were significantly reduced, but compared with the control group, the blood glucose level of the study group decreased more significantly, and the difference was statistically significant (*P* < 0.05), as shown in Figure 3.

### 3.6. Before and after Nursing, Renal Function Was Compared in the Two Groups

The renal function indicators of Scr and BUN between the two groups were not significantly different before breastfeeding (*P* > 0.05). The renal function indices of both groups were severely lowered after nursing, but the study group's renal function indexes declined more dramatically than those of the control group, and the difference was statistically significant.  Figure 4 shows the significance (*P*0.05).

## 4. Discussion

Patients with diabetic nephropathy who do not comprehend their condition and are concerned about their prognosis will experience negative emotions [7, 8]. As a consequence, patient nursing interventions are crucial. Previously, routine nursing treatments for diabetic nephropathy patients did not take into account the patient's emotional changes. They just did routine nurse interventions including medication counseling, life support, and health manual distribution. Despite the fact that they can achieve some effects, they have unsatisfactory outcomes [9–11]. The study carried out path-type health education for patients and can carry out various nursing interventions such as diet, psychology, and exercise, which can make up for the lack of conventional nursing care [12, 13].

Through patient education, pathway health education may successfully reduce blood sugar levels [14, 15]. By modifying the patient's diet and including aerobic activity, the sugar and salt intakes may be tightly regulated, thereby alleviating the symptoms of glomerular hyperfiltration, hyperperfusion, and hypertension [16–18]. Appropriate exercise greatly improves the patient's physique, immunological function, renal function, and microalbumin excretion level [19, 20]. The research's results suggested that both groups' blood glucose, liver, and kidney function indices decreased substantially after the intervention; however, the study group changed more significantly (*P*0.05) than the control group. The results suggested that path-based health education is more effective than standard care in controlling blood sugar and improving kidney function and that it is a safe and effective nursing practice. Patients with diabetic nephropathy often suffer from malnutrition, which is accompanied by noticeable changes in signs and symptoms, negatively affecting the patients' lives and quality of life [21]. Therefore, to improve patients' nutritional status, effective intervention measures should be developed to analyze the sodium, calorie, and protein content of food and to develop a reasonable plan to ensure balanced nutrition and to provide patients with the normal nutrition they require on a daily basis [22, 23]. The study's results indicated that although both groups' nutritional index values grew substantially after nursing, the study group's nutritional index values increased significantly (*P*0.05) more than those of the control group. When compared to typical nursing care, path-based health education seems to improve nutritional indicators more efficiently and has a good influence on illness recovery, according to the data. Disease management abilities for diabetic nephropathy patients should increase as a result of food intervention, which is favorable to improving patients' cognition. The results of the study showed that the GQOLI-74 and MUIS-A scores of the two groups were significantly increased, but compared with the control group, the study group changed more significantly (*P* < 0.05). The control group's awareness of drug treatment, basic knowledge, exercise, and diet was 79.4%, 78.9%, 73.4%, and 91.0%, respectively, and that of the study group was 90.3%, 96.4%, 92.8%, and 94.0%. Scholars' research results are consistent [24]. Studies have confirmed that path-based health education is more effective in improving disease management capabilities and improving disease awareness. Various biochemical markers in diabetic nephropathy patients will vary considerably, affecting the patient's normal life. Excess fat in the body can be removed, blood lipid metabolism can be improved, and endocrine function can be managed by path-type health education for the patient, all of which may lower the occurrence of renal menstruation. In summary, path-based health education is a novel form of nursing care that can enhance nutritional indicators and blood sugar and renal function and dramatically raise patients' knowledge of the condition, all of which can help them adhere to treatment better.

This nursing approach is practical to use and has a good clinical value.

## Figures and Tables

**Figure 1:** Comparison of nutritional indicators between the two groups before nursing.

**Figure 2:** Comparison of cognition between the two groups before and after nursing.

**Figure 3:** Changes of blood glucose levels in the two groups before and after nursing.

**Figure 4:** Comparison of renal function between the two groups before and after nursing.

**Table 1:** Comparison of GQOLI-74 and MUIS-A scores between the two groups before and after nursing$\left(\bar{x}\pm s\right)$.

Group	Number of cases	GQOLI-74 score		MUIS-A score	
		Before care	After care	Before care	After care
Control group	83	2.3 ± 0.2	3.5 ± 0.3	4.1 ± 0.8	3.5 ± 0.6
Research group	79	2.2 ± 0.3	4.9 ± 0.5	4.0 ± 0.9	2.0 ± 0.5
*T*	/	0.635	15.782	1.872	16.985
*P*	/	>0.05	>0.05	>0.05	<0.05

**Table 2:** Changes of biochemical indicators before and after nursing in the two groups$\left(\bar{x}\pm s\right)$.

Group	Number of cases	Total cholesterol (mmol/l)		Triglycerides (mmol/l)		Urea nitrogen (mmol/l)	
		Before care	After care	Before care	After care	Before care	After care
Control group	83	5.8 ± 1.8	5.6 ± 2.0	2.5 ± 1.2	2.5 ± 1.2	8.6 ± 4.1	7.8 ± 3.1
Observation group	79	5.5 ± 1.6	4.6 ± 1.5	2.4 ± 1.5	1.8 ± 1.1	8.5 ± 4.0	7.2 ± 2.2
*T*	/	1.635	15.724	0.862	14.035	0.785	18.426
*P*	/	>0.05	<0.05	>0.05	<0.05	>0.05	<0.05

## Data Availability

The data used to support the findings of this study are included within the article.

## References

[1] Wheeler D. C., Stefansson B. V., Batiushin M. (2020). The dapagliflozin and prevention of adverse outcomes in chronic kidney disease (DAPA-CKD) trial: baseline characteristics. *Nephrology, Dialysis, Transplantation*.

[2] Li J., Albajrami O., Zhuo M., Hawley C. E., Paik J. M. (2020). Decision algorithm for prescribing SGLT2 inhibitors and GLP-1 receptor agonists for diabetic kidney disease. *Clinical Journal of the American Society of Nephrology*.

[3] Ye X., Zhou X. J., Zhang H. (2019). Autophagy in immune-related renal disease. *Journal of Immunology Research*.

[4] Tucker K. L., Sheppard J. P., Stevens R. (2017). Self-monitoring of blood pressure in hypertension: a systematic review and individual patient data meta-analysis. *PLoS Medicine*.

[5] Cao X., Gong X., Ma X. (2019). Diabetic nephropathy versus diabetic retinopathy in a Chinese population: a retrospective study. *Medical Science Monitor*.

[6] Lo C., Toyama T., Wang Y. (2018). Insulin and glucose-lowering agents for treating people with diabetes and chronic kidney disease. *Cochrane Database of Systematic Reviews*.

[7] Kikuchi K., Saigusa D., Kanemitsu Y. (2019). Gut microbiome-derived phenyl sulfate contributes to albuminuria in diabetic kidney disease. *Nature Communications*.

[8] Geng X., Zhong D., Su L., Lin Z., Yang B. (2020). Preventive and therapeutic effect of _Ganoderma lucidum_ on kidney injuries and diseases. *Advances in Pharmacology*.

[9] Sulaiman M. K. (2019). Diabetic nephropathy: recent advances in pathophysiology and challenges in dietary management. *Diabetology and Metabolic Syndrome*.

[10] Tang S. C. W., Yu X., Chen H. C. (2020). Dialysis care and dialysis funding in Asia. *American Journal of Kidney Diseases*.

[11] Chen X., Yu J., Shi J. (2018). Management of diabetes mellitus with puerarin, a natural isoflavone from Pueraria lobata. *The American Journal of Chinese Medicine*.

[12] Lee Y. H. (2018). Socioeconomic differences among community-dwelling diabetic adults screened for diabetic retinopathy and nephropathy: the 2015 Korean Community Health Survey. *PLoS One*.

[13] Wang Y., Li M., Li C. (2020). Efficacy and safety of Shenkang injection as adjuvant therapy in patients with diabetic nephropathy: a protocol for systematic review and meta-analysis. *Medicine (Baltimore)*.

[14] Sevick M. A., Woolf K., Mattoo A. (2018). The Healthy Hearts and Kidneys (HHK) study: design of a 2 × 2 RCT of technology-supported self-monitoring and social cognitive theory-based counseling to engage overweight people with diabetes and chronic kidney disease in multiple lifestyle changes. *Contemporary Clinical Trials*.

[15] Jia Y., He J., Wang L. (2018). Dapagliflozin aggravates renal injury via promoting gluconeogenesis in db/db mice. *Cellular Physiology and Biochemistry*.

[16] Tan S. M., Ziemann M., Thallas-Bonke V. (2020). Complement C5a induces renal injury in diabetic kidney disease by disrupting mitochondrial metabolic agility. *Diabetes*.

[17] Koziolova N. A., Polyanskaya E. A., Surovtseva M. V., Karavaev P. G. (2018). Nonvalvular atrial fibrillation and diabetic nephropathy: epidemiology, prognosis, and choice of anticoagulant therapy. *Kardiologiia*.

[18] Regine I., Husain R. S. R. A., Aswathi R. P., Reddy D. R., Ahmed S. S. S. J., Ramakrishnan V. (2020). Asociacion entre el polimorfismo _rs1801282_ de PPAR *γ* con nefropatia diabetica y sensibilidad a la diabetes mellitus de tipo 2 en el sur de India y un metaanalisis. *Nefrología*.

[19] Kazawa K., Osaki K., Rahman M. M., Moriyama M. (2020). Evaluating the effectiveness and feasibility of nurse-led distant and face-to-face interviews programs for promoting behavioral change and disease management in patients with diabetic nephropathy: a triangulation approach. *BMC Nursing*.

[20] Cheema S., Maisonneuve P., Zirie M. (2018). Risk factors for microvascular complications of diabetes in a high-risk Middle East population. *Journal Diabetes Research*.

[21] Wang X., Liu Q., Kong D. (2020). Down-regulation of SETD6 protects podocyte against high glucose and palmitic acid-induced apoptosis, and mitochondrial dysfunction via activating Nrf2-Keap1 signaling pathway in diabetic nephropathy. *Journal of Molecular Histology*.

[22] Navarro-Flores E., Cauli O. (2020). Quality of life in individuals with diabetic foot syndrome. *Endocrine, Metabolic & Immune Disorders Drug Targets*.

[23] Li Y., Zhou H., Li Y. (2019). PTPN2 improved renal injury and fibrosis by suppressing STAT-induced inflammation in early diabetic nephropathy. *Journal of Cellular and Molecular Medicine*.

[24] Sinha N., Kumar V., Puri V. (2020). Urinary exosomes: potential biomarkers for diabetic nephropathy. *Nephrology (Carlton, Vic.)*.

